# The iron group transition-metal (Fe, Ru, Os) coordination of Se-doped graphitic carbon (Se@g-C_3_N_4_) nanostructures for the smart therapeutic delivery of zidovudine (ZVD) as an antiretroviral drug: a theoretical calculation perspective†

**DOI:** 10.1039/d3ra06885d

**Published:** 2023-11-21

**Authors:** Favour A. Nelson, Hitler Louis, Innocent Benjamin, Rawlings A. Timothy

**Affiliations:** a Computational and Bio-simulation Research Group, University of Calabar Calabar Nigeria louismuzong@gmail.com; b Department of Microbiology, University of Calabar Calabar Nigeria; c Department of Pure and Applied Chemistry, University of Calabar Calabar Nigeria; d Centre for Herbal Pharmacology and Environmental Sustainability, Chettinad Hospital and Research Institute, Chettinad Academy of Research and Education Kelambakkam 603103 Tamil Nadu India

## Abstract

This study employed density functional theory (DFT) computational techniques at the ωB97XD/def2svp level of theory to comprehensively explore the electronic behavior of Fe-group transition metal (Fe, Ru, Os) coordination of Se-doped graphitic carbon (Se@g-C_3_N_4_) nanosystems in the smart delivery of zidovudine (ZVD), an antiretroviral drug. The HOMO–LUMO results of the interactions show a general reduction in energy gap values across all complexes in the following order: ZVD_Se@C_3_N_4_ < ZVD_Ru_Se@C_3_N_4_ < ZVD_Fe_Se@C_3_N_4_ < ZVD_Os_Se@C_3_N_4_. ZVD_Se@C_3_N_4_ exhibits the smallest post-interaction band gap of 3.783 eV, while ZVD_Os_Se@C_3_N_4_ presents the highest energy band gap of 5.438 eV. Results from the corrected adsorption energy (BSSE) revealed that Os_Se@C_3_N_4_ and Ru_Se@C_3_N_4_ demonstrated more negative adsorption energies of −2.67 and −2.701 eV, respectively, pointing to a more favorable interaction between ZVD and these systems, thus potentially enhancing the drug delivery efficiency. The investigation into the drug release mechanism from the adsorbents involved a comprehensive examination of the dipole moment and the influence of pH, shedding light on the controlled release of ZVD. Additionally, investigating the energy decomposition analysis (EDA) revealed that ZVD_Ru_Se@C_3_N_4_ and ZVD_Fe_Se@C_3_N_4_ exhibited the same total energy of −787.7 kJ mol^−1^. This intriguing similarity in their total energy levels suggested that their stability was governed by factors beyond reactivity, possibly due to intricate orbital interactions. Furthermore, analyzing the bond dissociation energies showed that all systems exhibited negative enthalpy values, indicating that these systems were exothermic at both surface and interaction levels, thus suggesting that these processes emitted heat, contributing to the surrounding thermal energy.

## Abstract 2

This study employed DFT computational techniques at the ωB97XD/def2svp level of theory to explore the electronic behavior of Fe-group transition metal (Fe, Ru, Os) coordination of Se-doped graphitic carbon (Se@g-C_3_N_4_) nanosystems in the smart delivery of zidovudine (ZVD), an antiretroviral drug.

## 1 Introduction

Human immunodeficiency virus/acquired immunodeficiency syndrome (HIV/AIDS) stands as one of the most formidable global health challenges confronting humanity today.^1–3^ Since its initial discovery in May 1983, this viral scourge has inflicted weighty consequences on millions of individuals worldwide, causing severe repercussions in the realms of public health, societal structures, and the lives of individuals. HIV is an intricate medical condition that relentlessly undermines the immune system,^4–7^ diminishing its capacity to shield the body against infections and diseases. Due to the lack of a definitive cure for HIV/AIDS, substantial progress has been achieved in the development and deployment of antiretroviral drugs.^8^ When used judiciously, these medications can significantly extend the lifespans of those infected with the virus. HIV, classified as a retrovirus, employs a unique mechanism in which it converts its viral RNA genome into DNA using an enzyme known as reverse transcriptase.^9,10^ Antiretroviral drugs represent a distinct class of medications specifically designed to combat infections caused by HIV.^11^ They operate by impeding the replication and conversion of the viral RNA within the body, thereby retarding the progression of the virus. These antiretroviral drugs can be categorized based on the stage of the HIV life cycle that they target. Nucleoside analog reverse transcriptase inhibitors, such as zidovudine, lamivudine, stavudine, abacavir, emtricitabine, zalcitabine, dideoxycytidine, dideoxynosine, tenofovir disoproxil fumarate, and didanosine, function by integrating into the viral DNA,^12^ leading to chain termination. On the other hand, non-nucleoside analog reverse transcriptase inhibitors, including etravirine, delavirdine, efavirenz, and nevirapine, obstruct the binding capacity of the reverse transcriptase enzyme.^13–15^ Additionally, there are other classes of antiretroviral drugs, such as protease, fusion, and entry inhibitors, each with its distinctive mode of action.^16–20^

Recent research studies have unveiled a key challenge in the use of individual antiretroviral drugs as the virus' tendency to develop resistance over time.^21^ In a study by Niu *et al.*, a 2-dimensional phosphorene-based (DDS) delivery system is used for the delivery of zidovudine to increase its therapeutic effects.^22^ Consequently, researchers have developed a strategy involving the combination of two or more drugs to create a more potent antiretroviral therapy known as highly effective antiretroviral therapy (HAART).^23^ While HAART has proven effective in curbing resistance, it presents substantial drawbacks, particularly regarding cost and patient compliance, particularly in resource-limited settings where HIV prevalence is high. These concerns stem from the therapy's expense and the toxicity associated with frequent dosing.^24^ Addressing these challenges necessitates a reevaluation of drug delivery strategies. In a study by Ayub *et al.*, carbon nanocone oxide (ONC) is used as a drug carrier for zidovudine (ZVD) since they are efficient in delivering to the target site while reducing toxicity and generic accumulation, which are often related with intravenous traditional methods.^23,25^ Another promising avenue involves the use of nanoparticles, which offer precise drug targeting and reduce the need for frequent dosages. Nanoparticles encapsulate the drugs and deliver them directly to the specific target site within the body due to their diminutive size and polymeric composition.^26,27^ This approach allows medications to combat the virus more effectively, bypassing various metabolic processes that can compromise their efficiency before reaching the target site. Notably, studies by researchers such as Drake *et al.*^28^ have demonstrated the effectiveness of gold-encapsulated nanomaterials as a drug delivery system for HIV treatment, underscoring the potential of transition metals in enhancing antiretroviral drug delivery. Also, from researchers such as Bryant *et al.*, unmodified amino acid-functionalized borospherenes are used as a potential carrier for Lamivudine.^29^

In this research, the focus centers on tuning the electronic behavior of the studied systems by Fe-group transition metal coordination of Se-doped graphitic carbon for the effective delivery and controlled release of zidovudine within the framework of first-principles density functional theory (DFT) approach. The primary objective is to determine which of these systems offers the most effective drug delivery for zidovudine, while maintaining compatibility with human cells. The iron group transition metals, which include iron, ruthenium, and osmium,^30,31^ possess a unique set of outstanding qualities that make them compelling candidates for drug delivery applications. Their electronic structure, characterized by partially filled d-orbitals,^32^ leads to several key advantages. Firstly, these metals exhibit excellent electrical conductivity, allowing for the precise control of drug release from implanted devices or the use of electrical stimulation to enhance drug transport across biological barriers.^33^ Additionally, their strong magnetic properties, particularly in the case of iron, enable their utilization in magnetic resonance imaging (MRI) contrast agents, providing vital insights into tissue structures and functions. Their catalytic activity can be harnessed for chemical reactions relevant to drug synthesis, while their exceptional stability and resistance to corrosion make them suitable for implantable drug delivery systems.^34,35^ Furthermore, the mechanical properties of transition metals contribute to the reliability and durability of drug-delivery devices. Thus, the electronic characteristics of these metals, related to the valence and conduction band concept, underpin their potential for precision, safety, and efficiency in drug delivery, making them a promising choice for pharmaceutical innovations. According to a study by Pi *et al.*, graphitic carbon nitride has drawn a lot of attention in research due to its unique conduction band minimum (CBM = −1.3 eV) and valence band maximum (VBM = 1.4 eV).^36,37^ Furthermore, studies by Dennington *et al.* promoted the use of this material for photocatalysis processes.^38^ Although graphitic carbon nitride has some limitations, it is doped with Se to improve its properties alongside transitional metals in this study. This investigation holds promise in not only advancing the understanding of antiretroviral drug delivery, but also potentially providing an innovative solution to enhance the efficacy and accessibility of HIV/AIDS treatment.

## 2 Computational approach

### 2.1 DFT approach

The investigation detailed in this study hinged on the implementation of DFT calculations at the ωB97XD/def2svp level of theory. The primary objective was to evaluate the performance efficiency of Se-doped graphitic carbon (C_3_N_4_) nanostructures for the smart therapeutic delivery of Zidovudine, an antiretroviral drug. The optimization process for ZVD_Se@C_3_N_4_, incorporating additional doping with Fe, Os, and Ru, was meticulously executed using Gaussian 16 (ref. 39) and GaussView 6.0.16.^40^ The chosen computational method holds particular significance, as it facilitates an intricate exploration of molecular properties and interactions. This includes providing crucial insights into electronic structures, reactivity, and bonding mechanisms.^41,42^ Additionally, the study integrated a comprehensive set of objectives to effectively study the delivery of ZVD. This encompassed the analysis of frontier molecular orbitals (FMO) and natural bond orbital (NBO) analysis, along with density of states (DOS) assessments. These analyses collectively offered intricate insights into the electronic properties governing the behavior of the studied nanocomposites. For visualization of the highest molecular orbital and lowest unoccupied molecular orbital (HOMO–LUMO) isosurfaces, the chemcraft software^43^ was employed. Further scientific precision was introduced through the use of the Multiwfn package,^44^ enabling the exploration of the quantum theory of atoms-in-molecules (QTAIM) for insights into intermolecular interactions. A meticulous examination of non-covalent interactions (NCI) was conducted, providing insights into the non-bonding forces shaping the molecular assemblies. The visual dynamic simulation (VMD) software package^45^ was utilized for this purpose. The study extended its scope to encompass the UV excitation analysis, adsorption energy studies, and an in-depth exploration of sensor mechanisms. Furthermore, the effects of energy decomposition analysis and bond dissociation energy analysis were meticulously evaluated, along with molecular dynamic simulations to reveal the materials' responses to external perturbations. This comprehensive analytical framework collectively advances the understanding of the potential of Se-doped graphitic carbon (C_3_N_4_) nanostructures for the smart therapeutic delivery of Zidovudine.

### 2.2 Molecular dynamics simulation protocol

To evaluate the interaction between the adsorbate and the adsorbent, we used the Forcite Module on the Dassault Systèms BIOVIA software programme [cite]. Our study focused on the interaction between the adsorbate ZVD with Se@C_3_N_4_ and its doped systems of Fe, Os, and Ru. We used the NVT ensemble, a virtual laboratory that allowed us to examine the behavior of our molecular structures over a simulated time of 1 picosecond, equivalent to 1000 steps, and an arbitrary number seed of around 1.6 × 10^8^. The energy variables included a universal forcefield and charge.^46^ To add some randomness and excitement, we equipped our molecules with initial velocities that set their paths ablaze, and an arbitrary number seed of approximately 1.6 × 10^8^ to kindle the magic of this molecular performance. We employed cubic spline truncation for the atom-based summing of the van der Waals and electrostatic components, with a cutoff distance of 12.5 Å, spline width of 1 Å, and buffer width of 0.5 Å. The molecular symphony that unfolded during our simulation was vividly visualized and plotted using Origin Plot.

## 3 Results and discussion

### 3.1 Chemistry of 2D nanostructure

#### 3.1.1 Structural studies

Herein, the Density Functional Theory (DFT) method was utilized to calculate the bond lengths of various complexes, as demonstrated in Fig. 1 and 2. Specifically, investigating how the bond lengths change before and after the adsorption of the drug is shown in Table 1. For the ZVD_Fe_Se@C_3_N_4_ complex, prior to drug interaction, the bond length between the iron metal is marginally shorter than after adsorption, with a difference of 0.05319 Å. The bond between nitrogen and carbon remains relatively stable, showing little or no change, while the bond between carbon and selenium is slightly longer after drug interaction, although both values are approximately 1.9 Å. Notably, the bond between the metal ion and the hydrogen atom only forms after the adsorption process.^47,48^ This pattern is consistent across all other complexes, suggesting that they tend to develop additional bonds compared to the ordinary nanomaterial. After discussing the individual bonds within ZVD_Fe_Se@C_3_N_4_, it was observed that the bond lengths underwent minor changes upon drug addition, indicating the robustness of the complex, making it a promising candidate for drug delivery. Similar behavior is observed for ZVD_Os_Se@C_3_N_4_, with bond lengths before and after interaction showing comparable magnitudes. This pattern also extends to ZVD_Ru_Se@C_3_N_4_ and ZVD_Se@C_3_N_4_, where the bond lengths exhibit little variation after interaction. In summary, ZVD_Se@C_3_N_4_ exhibits the shortest bond lengths compared to the other complexes. Judging by bond length, it can be inferred that ZVD_Se@C_3_N_4_ is a more suitable candidate for drug delivery, as shorter bond lengths typically indicate stronger bonds. Therefore, the complexes can be ranked in terms of bond length increase as follows: ZVD_Se@C_3_N_4_ < ZVD_Fe_Se@C_3_N_4_ < ZVD_Os_Se@C_3_N_4_ < ZVD_Ru_Se@C_3_N_4_. Therefore, ZVD_Se@C_3_N_4_ emerges as the most promising nanomaterial for delivering zidovudine based on the bond length analysis of these complexes.

**Fig. 1:** An illustration of the drug target (zidovudine).

**Fig. 2:** A geometrical representation of the studied systems.

**Table 1:** Analysis of the nanocluster's chemistry calculated at the ωB97XD/def2svp level of theory

Systems	Bond labels	Bond lengths	
		Before interaction	After interaction
ZVD_Fe_Se@C_3_N_4_	Fe_55_–N_40_	2.17920	2.23239
	N_40_–C_14_	1.32925	1.34071
	C_14_–Se_54_	1.90176	1.88911
	Fe_55_–H_78_	—	1.65611
ZVD_Os_Se@C_3_N_4_	Os_55_–N_40_	2.3159	2.30041
	N_40_–C_14_	1.35015	1.35543
	C_14_–Se_54_	1.88872	1.88775
	Os_55_–O_56_	—	2.14502
ZVD_Ru_Se@C_3_N_4_	Ru_55_–N_40_	2.35625	2.32609
	N_40_–C_14_	1.34174	1.34258
	C_14_–Se_54_	1.90343	1.89748
	Ru_55_–H_78_	—	1.54090
ZVD_Se@C_3_N_4_	N_42_–C_16_	1.28962	1.28864
	C_16_–Se_54_	2.04277	1.95122

#### 3.1.2 Analysis of binding energy

Table 2 provides a comparative analysis of the binding energies for three different systems: Fe_Se@C_3_N_4_, Os_Se@C_3_N_4_, and Ru_Se@C_3_N_4_. These binding energies play a crucial role in understanding the stability and potential applications of these systems, particularly in the context of delivery.^49–51^ Looking at the data, it is evident that all three systems have negative binding energies, indicating attractive interactions between the molecules (Fe, Os, Ru) and the C_3_N_4_ substrate. However, the magnitude and sign of the binding energies differ significantly among the systems, which can provide insights into their respective characteristics. For Fe_Se@C_3_N_4_, the binding energy is approximately −5.4423 eV, indicating a moderately strong attractive interaction. This suggests that the Fe-containing system has a relatively stable bond with the C_3_N_4_ substrate, which could be advantageous for certain delivery applications. On the other hand, Os_Se@C_3_N_4_ exhibits a binding energy of approximately 5.4423 eV, which is of similar magnitude but opposite in sign to that of Fe_Se@C_3_N_4_. This positive binding energy suggests that there's a repulsive interaction between the Os-containing molecule and the C_3_N_4_ substrate. Such repulsion could have implications for applications where the controlled release or detachment of the molecule from the substrate is desired. Additionally, Ru_Se@C_3_N_4_ displays the most negative binding energy of approximately −27.211 eV, indicating a strong attractive interaction. The significantly higher binding energy of this system suggests a very stable bond with the C_3_N_4_ substrate, making it potentially suitable for applications where long-lasting and secure delivery is required. Overall, the comparative analysis of binding energies among these systems provides valuable insights into their stability and potential roles in delivery applications. The magnitude and sign of these energies can inform the design of systems tailored to specific delivery needs, whether it is controlled release, stability during transport, or long-term retention.

**Table 2:** The analysis of binding energy calculated at the ωB97XD/def2svp level of theory

Systems	*E*_surface_	*E*_M_	*E*_se@C_3_N_4__	Binding energy (eV)
Fe_Se@C_3_N_4_	−4607.6	−93.4	−4514	−5.4423
Os_Se@C_3_N_4_	−4604.7	−90.9	−4514	5.4423
Ru_Se@C_3_N_4_	−4608.9	−93.9	−4514	−27.211

#### 3.1.3 Vibrational stability

Table S1† displays the vibrational frequencies and their corresponding functional group assignments in various chemical systems. Vibrational frequencies are crucial for understanding how molecules behave.^52^ They offer insights into a molecule's stability, shape, and chemical characteristics.^53^ Upon exploring the vibrational stability provided in Table S1† concerning the reported functional groups and their frequencies, it was analyzed that the multiple vibrational frequencies of ZVD_Fe_Se@C_3_N_4_ were associated with different functional groups. For example, frequencies at 3787, 3776, and 3769 cm^−1^ corresponded to the asymmetric NH_2_ group, representing its stretching and bending vibrations in an asymmetric manner. Similarly, vibrations at 3649 and 3646 cm^−1^ were linked to the asymmetric NH group, while the features at 3634 and 3627 cm^−1^ indicated the symmetric NH_2_ stretching vibrations. In ZVD_Os_Se@C_3_N_4_, a symmetric OH stretching vibration appeared at 3921 cm^−1^. Asymmetric NH_2_ stretching vibrations occurred at 3786 and 3769 cm^−1^, and symmetric NH stretching vibrations were found at 3656, 3648, and 3644 cm^−1^. Symmetric NH_2_ stretching vibrations were observed at 3634 cm^−1^. The system also exhibited symmetric and asymmetric CH stretching vibrations at 3232 and 3176 cm^−1^, respectively. Additionally, asymmetric CH_3_ vibrations were detected at 3174 and 3141 cm^−1^, with symmetric CH_2_ and CH_3_ stretching vibrations at 3103, 3063, and 3054 cm^−1^. In ZVD_Ru_Se@C_3_N_4_, a symmetric OH stretching vibration was evident at 3938 cm^−1^. Asymmetric NH_2_ stretching vibrations were observed at 3792, 3791, and 3758 cm^−1^, while symmetric NH stretching vibrations occurred at 3658 and 3651 cm^−1^. Symmetric NH_2_ stretching was detected at 3627 cm^−1^. Additionally, symmetric CH stretching vibrations were present at 3273 cm^−1^, and asymmetric CH_3_ vibrations were observed at 3172, 3147, and 3058 cm^−1^. Symmetric CH_3_ stretching vibrations were found at 3058 cm^−1^, and a symmetric RuH stretching vibration appeared at 2283 cm^−1^. In the ZVD_Se@C_3_N_4_ system, asymmetric NH_2_ stretching vibrations were observed at 3794, 3789, and 3769 cm^−1^. Symmetric NH stretching vibrations occurred at 3652 cm^−1^, and symmetric NH_2_ stretching vibrations were detected at 3625 cm^−1^. Symmetric CH stretching vibrations were present at 3246 and 3199 cm^−1^, with asymmetric CH_3_ vibrations observed at 3169, 3148, and 3058 cm^−1^. Overall, these vibrational frequencies and assignments provide valuable insights into the chemical composition and structural stability of the studied systems.

### 3.2 UV-vis excitation analysis

The primary objective of this comprehensive analysis was to gain deeper insights into the various excitations exhibited by the numerous complexes that were rigorously examined in the course of our study, as presented in Table 3. The parameters that were meticulously scrutinized include excitation types, stabilization energy (*E*), wavelengths, oscillator strengths, transition contributions, and assorted assignments, all of which have been thoughtfully documented in Table 3. This analysis places great importance on the identification of exceptional systems, which are characterized by low stabilization energy, longer wavelengths, and higher oscillator strengths.^54,55^ These parameters as the basis for assessing the reactivity of the particles, guided by the fundamental energy–frequency relationship, were analyzed and expressed using eqn (1):

1 *E* = *hf*

Here, *E* represents the energy of the particle, *h* is the Planck constant (*h* = 6.626 × 10^−34^ J s), and *f* denotes the frequency of the particle. As per this formula, it is evident that energy is directly proportional to frequency. Simultaneously, it is well-established that frequency is inversely proportional to wavelength, as described in eqn (2):

2 *f* = *v*/*λ*

where *f* is the frequency, *v* is the speed of light, and *λ* is the wavelength. Hence, an increase in stabilization energy correlates with shorter wavelengths and enhanced reactivity of the particle. This foundational understanding serves as the cornerstone of our analytical approach. Upon close examination of the data presented in the table, it becomes evident that the interaction involving ZVD_Se@C_3_N_4_ exhibits the highest energy levels across all three excitation types. In the transition from the ground state (S_0_) to the first excited state (S_1_), this complex exhibits an energy of 1.6596 eV, while the transition to the second excited state (S_2_) boasts an energy level of 2.1082 eV. For the transition from S_0_ to the third excited state (S_3_), the energy climbs to 2.6512 eV. Remarkably, the corresponding wavelengths for these transitions are 747.05 nm, 588.11 nm, and 467.65 nm, which are notably the shortest among all of the data points. This observation implies that ZVD_Se@C_3_N_4_, although considered stable, is also highly reactive when compared to the other interactions investigated in this study. The oscillator strengths of these complexes span a range from 0.0 to 0.0149. Notably, the interaction ZVD_Se@C_3_N_4_ stands out with the highest percentage contribution of approximately 48% for the S_0_–S_1_ excitation type. Conversely, the S_0_–S_3_ excitation type from the interaction ZVD_Fe_Se@C_3_N_4_ exhibits the lowest percentage contribution, which amounts to 6.3%. Interestingly, ZVD_Fe_Se@C_3_N_4_ showcases the lowest stabilization energy among all three excitation types, with values of 0.4824 eV for S_0_–S_1_, 0.5747 eV for S_0_–S_2_, and 1.0425 eV for S_0_–S_3_. Correspondingly, the wavelengths for these transitions are 2570.35 nm, 2157.40 nm, and 1189.28 nm, respectively. Consequently, this leads us to conclude that ZVD_Fe_Se@C_3_N_4_ can be considered the most stable complex within the scope of this analysis, owing to its consistently low stabilization energy and relatively longer wavelengths.

**Table 3:** UV-vis excitation analysis calculated at the TD-DFT/ωB97XD/def2svp level of theory

Compound	Excitation type	Energy (eV)	Wavelength (nm)	Percentage contribution (%)	Oscillator strength	Transition (*f*)
ZVD_Fe_Se@C_3_N_4_	S_0_–S_1_	0.4824	2570.35	243 > 252 (8.5)	0.0002	H+7 → L−1
	S_0_–S_2_	0.5747	2157.40	236 > 252 (19.0)	0.0001	H+14 → L−1
	S_0_–S_3_	1.0425	1189.28	240 > 259 (6.3)	0.0000	H+10 → L−8
ZVD_Os_Se@C_3_N_4_	S_0_–S_1_	0.9594	1292.26	242 > 247 (35.6)	0.0014	H+3 → L−1
	S_0_–S_2_	1.1273	1099.86	241 > 247 (32.6)	0.0003	H+4 → L−1
	S_0_–S_3_	1.2660	979.37	240 > 247 (31.0)	0.0013	H+5 → L−1
ZVD_Ru_Se@C_3_N_4_	S_0_–S_1_	2.0024	619.17	243 > 246 (14.3)	0.0012	H+2 → L
	S_0_–S_2_	2.1636	573.04	244 > 246 (32.8)	0.0149	H+1 → L
	S_0_–S_3_	2.1816	568.32	244 > 246 (11.9)	0.0105	H+1 → L
ZVD_Se@C_3_N_4_	S_0_–S_1_	1.6596	747.05	237 > 238 (48.0)	0.0001	H → L
	S_0_–S_2_	2.1082	588.11	236 > 238 (46.1)	0.0004	H+1 → L
	S_0_–S_3_	2.6512	467.65	237 > 240 (31.9)	0.0011	H → L−2

### 3.3 Electronic property investigation

#### 3.3.1 Chemical reactivity descriptors

The energy gap, defined as the energy difference between the highest occupied molecular orbital (HOMO) and the lowest unoccupied molecular orbital (LUMO),^56,57^ serves as a crucial indicator of the reactivity of chemical complexes as graphically illustrated in Fig. 3. In the context of this study, this parameter offers valuable insights into the reactivity of the complexes under investigation, as presented in Table 4. Analyzing the data presented in Table 4, it becomes evident that the energy gap values, measured before any interaction with the drug, exhibited an ascending order: Ru_Se@C_3_N_4_ < Os_Se@C_3_N_4_ < Se@C_3_N_4_ < Fe_Se@C_3_N_4_. Remarkably, Ru_Se@C_3_N_4_ possessed the smallest energy gap, measuring at 5.098 eV, while Fe_Se@C_3_N_4_ boasts the most extensive energy gap, reporting at 6.934 eV. These energy gap values are particularly noteworthy because they convey the stability and reactivity of these complexes.^58,59^ An energy gap value exceeding 5.0 eV generally signifies limited electron transfer and reduced reactivity, indicating that these complexes can be considered stable and less prone to chemical reactions. Post-interaction, a general reduction in energy gap values was observed across all the complexes, following this order: ZVD_Se@C_3_N_4_ < ZVD_Ru_Se@C_3_N_4_ < ZVD_Fe_Se@C_3_N_4_ < ZVD_Os_Se@C_3_N_4_. Notably, ZVD_Se@C_3_N_4_ exhibits the smallest post-interaction band gap, measuring at 3.783 eV, while ZVD_Os_Se@C_3_N_4_ presents the highest energy band gap, amounting to 5.438 eV. This intriguing trend reveals a pivotal aspect of the complexes' compatibility with the drug. Complexes that initially possessed larger band gaps tended to experience a reduction in their band gap values following interaction with the drug, indicating an increased reactivity and a propensity for electron transfer.^60^ Conversely, complexes with smaller initial band gaps demonstrated an increase in their band gap values post-interaction, suggesting a reduced reactivity and a reluctance to engage in chemical reactions.^61^ Thus, the analysis of the band gap values offers valuable insights into the compatibility of these complexes with the drug, shedding light on their reactivity and stability in the presence of the drug. Remarkably, based on this band gap analysis, ZVD_Se@C_3_N_4_ continues to emerge as the most promising candidate for the delivery of zidovudine, closely followed by ZVD_Ru_Se@C_3_N_4_. To back up this explanation, the systems were optimized using the PBEO hybrid density functional, and the energy gaps were calculated and recorded in Table S6 of the ESI.† The values of the energy from the PBE0 method are much smaller compared to the ωB97XD/def2svp level of theory, but still agrees with the explanation given above, as ZVD_Se@C_3_N_4_ still tends to possess the smallest energy gap of −0.024 eV. In addition to the valuable insights gained from band gap analysis, it is essential to consider the ionization potential (IP) and electron affinity (EA) when evaluating the reactivity and stability of chemical complexes in their specific environmental contexts. A high ionization potential signifies that a complex is inherently stable and exhibits reluctance to engage in chemical reactions within a given environment.^62^ Conversely, a high electron affinity indicates that the complex possesses a strong inclination to form bonds and engage in the transfer of electrons, suggesting its readiness to participate in chemical interactions.^63^ Examining these parameters in our study, we find that ZVD_Ru_Se@C_3_N_4_ displays the smallest ionization potential, measured at 5.812 electronvolts (eV). This result implies that ZVD_Ru_Se@C_3_N_4_ is predisposed to readily release electrons, showcasing its heightened reactivity and potential for electron donation compared to the other complexes under investigation. On the other hand, ZVD_Se@C_3_N_4_ exhibits the highest electron affinity, measuring approximately 2.327 eV. This noteworthy value suggests that ZVD_Se@C_3_N_4_ possesses a remarkable propensity to accept electrons, positioning it as an ideal candidate for forming bonds and participating in electron transfer processes with other chemical species. These findings reinforce our earlier conclusion regarding ZVD_Se@C_3_N_4_'s exceptional suitability for the delivery of zidovudine. Its combination of properties, including a reduced band gap, high electron affinity, and the highest electron affinity among the complexes, reaffirms its standing as the prime choice for facilitating the controlled and efficient delivery of zidovudine. Furthermore, the phenomenon of electronegativity warrants consideration in our analysis. Electronegativity generally increases following interactions with zidovudine. Notably, ZVD_Se@C_3_N_4_ exhibits the most substantial increase in electronegativity, measuring at 0.264. This remarkable rise underscores ZVD_Se@C_3_N_4_'s ability to attract electrons closer to itself in chemical interactions, ultimately leading to the development of polarity and a higher dipole moment within the complex. In summary, our comprehensive assessment of the ionization potential, electron affinity, and electronegativity collectively bolsters the assertion that ZVD_Se@C_3_N_4_ remains the optimal nanomaterial for the precise delivery of zidovudine. Its exceptional combination of properties, coupled with the demonstrated tendency to increase electronegativity upon interaction with zidovudine, underscores its capacity to establish favorable chemical interactions and enhance the drug delivery process with precision and efficiency.

**Fig. 3:** A graphical demonstration of the HOMO–LUMO isosurfaces for the studied systems.

**Table 4:** The analysis of various discussed chemical quantum descriptors calculated at the ωB97XD/def2svp level of theory

Systems	HOMO/eV	LUMO/eV	*E*_gap_/eV	IP	EA	*σ*	*Π*	*μ*	*χ*	*E*_FL_
Fe_Se@C_3_N_4_	−8.287	−1.353	6.934	8.287	1.353	0.144	3.467	−4.820	3.351	4.820
Os_Se@C_3_N_4_	−6.269	−0.562	5.706	6.269	0.562	0.175	2.853	−3.416	2.044	3.416
Ru_Se@C_3_N_4_	−5.914	−0.816	5.098	5.914	0.816	0.196	2.549	−3.365	2.221	3.365
Se@C_3_N_4_	−6.593	−0.480	6.113	6.593	0.480	0.164	3.056	−3.536	2.046	3.536
ZVD_Fe_Se@C_3_N_4_	−6.104	−1.155	4.949	6.104	1.155	0.202	2.474	−3.629	2.662	3.629
ZVD_Os_Se@C_3_N_4_	−6.502	−1.063	5.438	6.502	1.063	0.184	2.719	−3.782	2.631	3.782
ZVD_Ru_Se@C_3_N_4_	−5.812	−0.916	4.896	5.812	0.916	0.204	2.448	−3.364	2.311	3.364
ZVD_Se@C_3_N_4_	−6.109	−2.327	3.783	6.109	2.327	0.264	1.891	−4.218	4.704	4.218

#### 3.3.2 Second order perturbation energy analysis

NBO analysis is a powerful tool in chemistry that employs second-order perturbation energy as a benchmark for understanding the distribution of electrons within molecular systems.^64,65^ This analysis is instrumental in elucidating the movement of electrons from donor to acceptor orbitals, shedding light on the intricacies of chemical interactions. Second-order perturbation energy represents the energy required for the delocalization of electrons.^66,67^ It plays a pivotal role in the analysis of electron movements and is a cornerstone of NBO analysis. Through this analysis, it can dissect how electrons shift between different molecular orbitals, a crucial aspect in understanding chemical reactivity. The interaction ZVD_Fe_Se@C_3_N_4_ exhibits the highest perturbation energy, measuring at an impressive 25.67 kcal mol^−1^, as shown in Table 5. Following closely is its surface counterpart, Fe_Se@C_3_N_4_, with an energy value of 24.25 kcal mol^−1^. Remarkably, the same orbital interactions are observed for both the surface and the interaction, underscoring the consistency of these interactions across different conditions. Examining the complexes, Fe_Se@C_3_N_4_ and ZVD_Fe_Se@C_3_N_4_, we find that they exhibit πC_16_–N_41_ orbital interactions, with energies of 6.96 kcal mol^−1^ and 14.80 kcal mol^−1^, respectively. The second interaction involves LP(1)N_38_ donating to LP(6)Fe_55_, with energies of 17.29 kcal mol^−1^ and 10.87 kcal mol^−1^ for the surface and interaction, respectively. This analysis highlights an important trend: the energy required for electron transfer increases in the interaction, signifying a greater demand for energy when transferring electrons from the respective donors to their acceptors. These transitions in ZVD_Fe_Se@C_3_N_4_ and its surface are characterized as π–π* and LP–LP. These transitions are indicative of weak covalent bonds and the presence of lone pairs, providing valuable insights into the nature of the chemical bonds formed in this system. Moving on to the ZVD_Os_Se@C_3_N_4_ system, we find a slightly lower perturbation energy of 4.11 kcal mol^−1^ in the interaction, compared to the surface energy of Os_Se@C_3_N_4_, which is 5.93 kcal mol^−1^. The transitions in this case involve σ-LP* and π-LP*. These transitions suggest distinct types of electron movements, each associated with its own energy demand, contributing to the complexity of the chemical interactions within this system. Interestingly, the complexes containing the ruthenium metal exhibit the lowest perturbation energy values on the table. The surface has an energy of 1.72 kcal mol^−1^, and the interaction has a slightly higher value of 1.92 kcal mol^−1^. The transitions in this case are characterized as σ-LP*, with energy values of 1.16 kcal mol^−1^ for the surface and 0.56 kcal mol^−1^ for the interaction, as well as 0.91 kcal mol^−1^ for the surface and 1.01 kcal mol^−1^ for the interaction. These values indicate that the ruthenium complexes involve a distinct and comparatively weaker electron transfer process compared to the other systems.

**Table 5:** The analysis of the natural bond orbital (NBO) calculated at the ωB97XD/def2svp level of theory

Systems	Donor	Occ	Acceptor	Occ	*E* ^2^/kcal mol^−1^	*E* ^2^ (total)/kcal mol^−1^	*E*(*j*) − *E*(*I*)	*F* (*I*, *j*)	Hybrid	Atomic orbital
Fe_Se@C_3_N_4_	πC_16_–N_41_	0.988	π*C_14_–Se_54_	0.034	6.96	24.25	0.35	0.065	Spd^43%^	s(32.91%) p 2.04(67.02%) d 0.00(0.07%)
	LP(1)N_38_	0.946	LP(6)Fe_55_	0.054	17.29		0.52	0.125	—	s(27.20%) p 2.67(72.71%) d 0.00(0.09%)
Os_Se@C_3_N_4_	σC_14_–Se_54_	0.903	LP*(6)Os_55_	0.031	2.27	5.93	1.38	0.071	Spd^56%^	s(0.13%) p 99.99(99.74%) d 0.92(0.12%)
	πC_1_–N_38_	0.989	LP*(4)Os_55_	0.193	3.64		0.74	0.068	Spd^38%^	s(34.31%) p 1.91(65.56%) d 0.00(0.13%)
Ru_Se@C_3_N_4_	σC_1_–N_38_	0.990	LP*(4)Ru_55_	0.029	1.16	1.72	0.92	0.048	Spd^39%^	s(34.62%) p 1.89(65.27%) d 0.00(0.12%)
	σC_1_–N_37_	0.989	LP*(7)Ru_55_	0.029	0.56		1.19	0.033	41	s(35.32%) p 1.83(64.57%) d 0.00(0.11%)
Se@C_3_N_4_	σC_16_–Se_54_	0.989	π*C_15_–N_44_	0.023	2.47	2.91	1.66	0.081	Spd^53%^	s(35.18%) p 1.84(64.72%) d 0.00(0.10%)
	LP(2)N_45_	0.809	π*C_14_–Se_54_	0.338	0.44		0.23	0.014	Spd^62%^	s(0.13%) p 99.99(99.72%) d 1.05(0.14%)
ZVD_Fe_Se@C_3_N_4_	πC_16_–N_41_	1.799	π*C_14_–Se_54_	1.963	14.80	25.67	0.37	0.077	54	s(31.29%) p 2.19(68.60%) d 0.00(0.11%)
	LP(1)N_38_	1.776	LP(6)Fe_55_	0.332	10.87		0.47	0.065	—	s(26.32%) p 2.80(73.64%) d 0.00(0.04%)
ZVD_Os_Se@C_3_N_4_	σC_14_–Se_54_	1.971	LP*(6)Os_55_	0.116	1.44	4.11	1.42	0.041	38	s(34.24%) p 1.92(65.64%) d 0.00(0.12%)
	σC_1_–N_38_	1.977	LP*(4)Os_55_	0.103	2.67		1.24	0.053	39	s(34.49%) p 1.90(65.39%) d 0.00(0.12%)
ZVD_Ru_Se@C_3_N_4_	σC_1_–N_38_	1.979	LP*(4)Ru_55_	0.096	0.91	1.92	1.15	0.029	39	s(35.12%) p 1.84(64.76%) d 0.00(0.11%)
	σC_15_–Se_54_	1.982	LP*(7)Ru_55_	0.033	1.01		1.31	0.033	39	s(38.62%) p 1.59(61.26%) d 0.00(0.12%)
ZVD_Se@C_3_N_4_	σC_16_–Se_54_	1.979	σ*C_15_–N_44_	0.047	4.96	5.68	1.66	0.082	53	s(35.28%) p 1.83(64.61%) d 0.00(0.11%)
	LP(1)N_45_	1.794	π*C_14_–Se_54_	0.121	0.72		1.01	0.024	45	s(29.43%) p 2.40(70.48%) d 0.00(0.10%)

#### 3.3.3 Density of states (DOS) analysis

DOS holds a paramount position in the investigation of drug delivery applications by providing an elaborate comprehension of the electronic structure and energy distribution within materials employed in sensing devices.^64,65^ By providing a detailed mapping of the energy levels accessible to electrons, DOS offers comprehensive insights into the electronic structure and energy distribution within materials, influencing their electrical conductivity. This influence becomes particularly crucial when considering the delivery of targeted drug species, such as the antiretroviral drug zidovudine (ZVD) used in HIV treatment. The alterations induced by specific drug molecules on DOS can lead to changes in the electronic properties of the material, including shifts in the band gap and variations in carrier concentration.^68,69^ These changes, in turn, directly correlate with modifications in electrical conductivity, forming the foundational basis for the detection and quantification of the targeted drug species. Consequently, DOS has become an indispensable tool for understanding drug-delivery phenomena, facilitating the strategic design, and optimization of delivery materials to enhance sensitivity and selectivity. In the context of this study, which explores systems incorporating ZVD_Fe_Se@C_3_N_4_, ZVD_Os_Se@C_3_N_4_, ZVD_Ru_Se@C_3_N_4_, and ZVD_Se@C_3_N_4_, the insights gained through DOS elucidate the electronic structures and energy distribution profiles of incorporated dopants, including Fe, Os, and Ru. Notably, Fe emerges as a key element, evidenced by its prominent manifestation in Fig. 4 and the relatively narrower energy gap of −0.4 to −0.6 eV computed for the ZVD_Fe_Se@C_3_N_4_ system. This observation implies heightened reactivity, elevated conductivity, and amplified selectivity of the examined surface in effectively delivering ZVD within the human body. Conversely, the contribution of Os is linked to the introduction of additional orbitals during the decoration process. These orbitals are postulated to facilitate mediating interactions with drug molecules, thereby enhancing the material's delivery capabilities. The outcomes underscore the profound potential of the studied systems, stimulated with Fe, Os, and Ru dopants, in advancing the domain of drug delivery. The revelatory understanding of electronic structures and energy distributions bestowed by DOS accentuates the tailored reactivity and conductivity of these surfaces, magnifying their efficacy in delivering ZVD.

**Fig. 4:** Illustrations of the total, partial, and overlap density of states for the various studied systems.

### 3.4 Visual studies

#### 3.4.1 Analysis of the quantum theory of atoms-in-molecules (QTAIM)

Bader's theory of topology analysis provides a vital parameter to study intermolecular and intramolecular interactions, which is known as the QTAIM. QTAIM helps us understand interactions between molecules.^70,71^ These parameters are associated with quantum topological functions and include the following: electron density (*ρ*(*r*)), Laplacian of electron density (∇^2^(*r*)), Lagrangian kinetic energy (*G*(*r*)), Hamiltonian kinetic energy (*K*(*r*)), potential energy density (*V*(*r*)), energy density (*H*(*r*)), Eigen values of Hessian (*λ*_1_ and *λ*_2_), ellipticity of electron density (*ε*), and electron localization function (ELF). The presence of bond critical points (BCPs) is indicative of chemical bonds like hydrogen bonds, as demonstrated in Fig. 5 and S1 of the ESI.† Identifying BCPs enhances the calculation of various topological parameters. According to existing literature,^72^ higher values of electron density (*ρ*(*r*)) represent stronger chemical bonds, while lower values depict weaker chemical bonds.^73^Table 6 illustrates that the highest *ρ*(*r*) value is observed in the C_1_–O_5_ bond (0.575 a.u.) in ZVD_Fe_Se@C_3_N_4_, the Ru_55_–N_40_ bond (0.466 a.u.) in Ru_Se@C_3_N_4_, the Se_54_–C_14_ bond (0.333 a.u.) in Ru_Se@C_3_N_4_, and the Se_54_–C_6_ bond (0.392 a.u.) in ZVD_Se@C_3_N_4_ complexes, indicating chemical bonds between the drug carrier and drug molecule. Negative values of ∇^2^(*r*) and *H*(*r*) signify strong covalent interactions, positive ∇^2^(*r*) values and negative *H*(*r*) values indicate medium interactions, while both positive values (∇^2^(*r*) > 0, *H*(*r*) > 0) denote weak (non-covalent) interactions.^74^ It is worth noting that bonds attached to the drug carrier generally show positive ∇^2^(*r*) values and negative *H*(*r*) values, demonstrating medium interactions, except for the Se_54_–C_14_ bond, which has both negative ∇^2^(*r*) (−0.549 a.u.) and *H*(*r*) (−0.453 a.u.). After the drug carriers interact with the drug molecule, bonds Se_54_–C_14_, Se_54_–C_6_, and Se_54_–O_5_ exhibit negative ∇^2^(*r*) and *H*(*r*) values, indicating strong covalent interactions in the ZVD_Se@C_3_N_4_ complex. Similarly, bonds Os_55_–O_5_ and Se_54_–O_5_ in ZVD_Os_Se@C_3_N_4_ also display both negative ∇^2^(*r*) and *H*(*r*) values, indicating strong covalent interaction. However, the Fe_55_–N_38_ and C_1_–O_5_ bonds in ZVD_Fe_Se@C_3_N_4_ have both positive ∇^2^(*r*) and *H*(*r*) values, signifying non-covalent interaction. Also, the Ru_55_–O_5_ bond has a positive ∇^2^(*r*) and negative *H*(*r*) value, indicating medium interaction in ZVD_Ru_Se@C_3_N_4_.

**Fig. 5:** Plots illustrating the paths and BCPs for the studied systems.

**Table 6:** The analysis of QTAIM parameters

System	Interaction	BCPs	*P*(*r*)	∇^2^*ρ*(*r*)	*G*(*r*)	*V*(*r*)	*H*(*r*)	−*G*(*r*)/*V*(*r*)	ELF	LOL	*λ*_1_	*λ*_2_	*λ*_3_	*ε*
Fe_Se@C_3_N_4_	Fe_55_– N_46_	105	0.207	0.539	0.155	−0.175	−0.199	−0.886	0.773	0.224	0.807	−0.124	−0.144	0.16028
	Se_54_–C_16_	86	0.145	0.329	0.772	−0.725	0.473	−1.065	0.927	0.242	−0.766	−0.817	0.487	0.06647
Os_Se@C_3_N_4_	Os_55_–N_50_	85	0.279	0.105	0.268	−0.275	−0.668	−0.975	0.711	0.216	0.357	0.119	−0.182	−6.0996
	Os_55_–N_39_	112	0.279	0.993	0.258	−0.269	−0.104	−0.959	0.762	0.223	−0.318	0.121	−0.182	−6.2926
Ru_Se@C_3_N_4_	Ru_55_–N_40_	103	0.466	0.209	0.553	−0.582	−0.289	−0.950	0.897	0.238	0.294	−0.493	−0.352	0.39773
	Se_54_–C_14_	85	0.333	−0.549	0.316	−0.769	−0.453	−0.411	0.679	0.593	−0.681	0.740	−0.608	0.12047
Se@C_3_N_4_	Se_54_–C_14_	95	0.109	0.247	0.311	−0.758	−0.447	−0.410	0.836	0.691	0.256	−0.131	−0.122	0.07815
	N_46_–N_38_	107	0.180	0.843	0.177	−0.144	0.335	−1.229	0.386	0.167	0.116	−0.159	−0.156	0.02375
ZVD_Fe_Se@C_3_N_4_	Fe_55_–N_38_	114	0.139	0.511	0.114	−0.100	0.139	−1.140	0.398	0.169	−0.959	−0.136	0.743	0.41875
	C_1_–O_5_	166	0.575	0.229	0.461	−0.349	0.112	−1.321	0.129	0.103	−0.698	0.341	0.202	−1.2046
ZVD_Os_Se@C_3_N_4_	Os_55_–O_5_	8	0.191	−0.115	0.277	−0.288	−0.288	−0.962	0.999	0.998	−0.384	−0.384	−0.384	0.00002
	Se_54_–O_5_	6	0.117	−0.511	0.708	−0.128	−0.128	−5.531	0.999	0.999	−0.170	−0.170	−0.170	0.00001
ZVD_Ru_Se@C_3_N_4_	Ru_55_–O_5_	170	0.151	0.249	0.134	−0.205	−0.714	−0.654	0.460	0.480	−0.219	−0.208	0.675	0.05371
	Se_54_–C_14_	210	0.299	−0.141	0.328	−0.417	−0.385	−0.787	0.993	0.921	−0.125	0.106	−0.122	0.02567
ZVD_Se@C_3_N_4_	Se_54_–C_6_	25	0.392	−0.175	0.435	−0.438	−0.438	−0.993	0.999	0.993	−0.543	−0.604	−0.603	0.00072
	Se_54_–O_5_	27	0.117	−0.510	0.642	−0.128	−0.128	−5.016	0.999	0.999	−0.170	−0.170	−0.170	0.00001

Furthermore, low values of ellipticity of electron density (*ε*) correspond to structural stability, whereas higher *ε* values correlate with structural instability of the interactions. Notably, *ε* values after the drug carrier interacts with the drug molecule are generally very low, indicating structural stability, except for the Fe_55_–N_38_ bond (0.41875 a.u.) in ZVD_Fe_Se@C_3_N_4_, which has the highest *ε* value, making it relatively unstable. According to the literature,^75^ ELF values below 0.5 a.u. represent delocalized electrons. It can also be observed that after the interaction of the drug carrier with the drug molecule, all the complexes have localized electrons due to ELF values above 0.5 a.u., except for the Fe_55_–N_38_ and C_1_–O_5_ bonds, which have ELF values of 0.398 a.u. and 0.129 a.u., indicating a high tendency of delocalized electrons in ZVD_Fe_Se@C_3_N_4_. Based on the reported literature,^76^ positive values of *λ*_2_ correspond to steric repulsion, while negative values indicate attractive forces. Table 6 reveals that only the C_1_–O_5_ bond (0.341 a.u.) in ZVD_Fe_Se@C_3_N_4_ and the Se_54_–C_14_ bond (0.106 a.u.) in ZVD_Ru_Se@C_3_N_4_ demonstrate steric repulsion, while all other interactions reflect negative *λ*_2_ values, implying that the interactions within the BCPs are primarily stabilizing interactions due to attractive forces.

#### 3.4.2 Reduced density gradient analysis (RDG)

The concept of Reduced Density Gradient (RDG) analysis, also known as non-covalent interactions (NCI), holds great significance in various fields like drug development, materials science, and biochemistry.^77^ Investigating the interactions between molecules that do not involve electron exchange is especially important when covalent bonding is absent. Despite being weaker, non-covalent interactions play a substantial role in biological, chemical, and physical processes occurring within molecules. In the area of drug discovery, researchers employ RDG analysis to explore how medicinal molecules interact with target proteins, facilitating the development of more effective and specific medications.^78^ The primary categories of non-covalent interactions encompass electrostatic interactions, van der Waals forces, hydrogen bonding, and hydrophobic interactions.^79^ The computationally visualized RDG map serves as a tool for comprehending intramolecular and intermolecular interactions within and between the systems under study. This map depicts various distinct regions enabled by the iso-surfaces it generates, including van der Waals contacts, steric repulsion, and strong attractive forces. In Fig. 6, the colors of the iso-surfaces can be interpreted as follows: green iso-surfaces represent non-directional attraction resulting from weak interactions, specifically van der Waals dispersion forces.^80^ Conversely, red iso-surfaces signify robust interactions primarily driven by steric repulsion, although they exert a significant influence on the reactivity and conformation of ions and molecules. On the iso-surfaces of the drug carriers, it is notable that the area around the Metals is characterized by strong interaction due to steric repulsion. It can also be seen that upon interaction of the drug carrier with the drug molecule, the green iso-surfaces are scattered on the system, being more intense around the site with the drug molecule. This indicates that the drug molecule and the delivery systems are characterized by non-directional attraction resulting from van der Waals dispersion forces. However, the NCI analysis is in agreement with the QTAIM analysis, as the systems are mostly characterized by non-directional attractive forces.

**Fig. 6:** Plots demonstrating the non-covalent interactions of the studied systems.

### 3.5 Molecular dynamic studies

Molecular dynamics simulations represent an invaluable arsenal within the realm of computational chemistry.^81^ They allow us to peer into the intricate dance of atoms and molecules over time, offering a comprehensive understanding of their behavior and interactions within biological systems during delivery.^82^ This analytical approach involves scrutinizing a variety of energy metrics, such as initial energies, final energies, average energies, and their associated standard deviations, in order to unravel the secrets of molecular stability and interaction with biological systems.^83,84^ The following discussion delves into the intriguing dynamics of different systems, each interacting with zidovudine, while considering various sites of adsorption. At the forefront of this investigation are four different systems, each bearing a unique site of adsorption for zidovudine: ZVD_Se@C_3_N_4_, ZVD_Ru_Se@C_3_N_4_, ZVD_Fe_Se@C_3_N_4_, and ZVD_Os_Se@C_3_N_4_. These systems are visually represented in the accompanying Fig. 7, and the extracted data are presented in Table S2 of the ESI.† Starting with ZVD_Fe_Se@C_3_N_4_, we observe an initial energy of 2007.364 kcal mol^−1^, which moderately increases to 2013.267 kcal mol^−1^ in the final energy assessment. This augmentation suggests a favorable interaction with zidovudine. The average energy for this system registers at 2011.286 kcal mol^−1^, although it is accompanied by a relatively high standard deviation of 3.652 kcal mol^−1^. Conversely, ZVD_Os_Se@C_3_N_4_, ZVD_Ru_Se@C_3_N_4_, and ZVD_Se@C_3_N_4_ exhibit total energy values that follow a similar trend, with final energies slightly lower than initial energies. The average energies for these systems remain closely aligned with their respective final energies, indicating relative stability. Furthermore, the standard deviations of these systems suggest that the energies remain relatively consistent throughout the simulation before the molecules bond with zidovudine. In the case of Fe_Se@C_3_N_4_, the total energy experiences a slight decrease from 1512.439 kcal mol^−1^ to 1511.88 kcal mol^−1^. The average energy is recorded at 1509.189 kcal mol^−1^, accompanied by a standard deviation of 2.313 kcal mol^−1^, indicating some fluctuations during the simulation. The other systems exhibit analogous trends, with final energies slightly below their initial counterparts and relatively stable average energies. The standard deviations for these systems are also relatively low, indicating consistent behavior during the interaction. The potential energy, which constitutes the dominant component of the total energy, plays a pivotal role in determining the systems' stability and their interactions with zidovudine. The decrease in potential energy from the initial to the final values suggests that these systems undergo favorable energy changes, resulting in the formation of stable configurations with zidovudine. Notably, in the case of ZVD_Fe_Se@C_3_N_4_, the initial potential energy is significantly higher at 1930.972 kcal mol^−1^, in contrast to the final potential energy of 1158.973 kcal mol^−1^. This substantial decrease underscores the system's favorable interaction with zidovudine, culminating in a more stable configuration. The average potential energies for the various systems exhibit a similar trend, although the standard deviations indicate some variations, likely stemming from dynamic changes and fluctuations during the simulations. Although contributing a smaller fraction to the total energy, the kinetic energy provides insights into the motion and thermal behavior of the systems. Calculated temperatures based on the kinetic energy reveal variations among the different systems. Higher temperatures generally indicate more energetic particle motion. For instance, ZVD_Fe_Se@C_3_N_4_ exhibits an initial temperature of 298 K, which increases significantly to 3332.539 K in the final assessment. These temperature variations reflect the diverse dynamics and thermal behaviors of the systems. In summary, the calculated energies shed light on the stability and interactions of the different adsorption sites with zidovudine. The slight decrease in total energy from initial to final assessments suggests favorable interactions and increased stability. The low standard deviations for the average energies indicate consistent behavior and minimal fluctuations during the simulations. These findings contribute significantly to our technical understanding of how systems with various adsorption sites interact favorably with zidovudine, hinting at their potential utility in drug delivery applications.

**Fig. 7:** A graphical representation of the molecular dynamic simulations for the studied systems.

### 3.6 Adsorption energy analysis corrected at BSSE

Table 7 offers a comprehensive insight into the adsorption energies corrected (BSSE) of ZVD drug molecules across various systems, including Fe_Se@C_3_N_4_, Os_Se@C_3_N_4_, Ru_Se@C_3_N_4_, and Se@C_3_N_4_. These adsorption energies play a pivotal role in determining the efficacy of drug binding to these systems, thereby influencing the overall drug delivery process.^85,86^ Additionally, the pH-dependent drug release values provide valuable information about how pH conditions can impact the release of the drug from these systems.^87,88^ Examining the adsorption energies, it is notable that all of the systems exhibit negative values, indicating a favorable adsorption of ZVD onto these substrates. However, the magnitude of these energies varies significantly among the systems. ZVD_Fe_Se@C_3_N_4_ stands out with an adsorption energy of −1.561 eV, suggesting a weaker interaction between ZVD and this system. This weaker binding implies that ZVD_Fe_Se@C_3_N_4_ might be less conducive for efficient drug delivery. On the contrary, ZVD_Os_Se@C_3_N_4_ and ZVD_Ru_Se@C_3_N_4_ demonstrate more negative adsorption energies of −2.67 and −2.701 eV, respectively. These stronger adsorption energies point to a more favorable interaction between ZVD and these systems, potentially enhancing the efficiency of drug delivery. In contrast, ZVD_Se@C_3_N_4_ shows a moderate adsorption energy of −1.945 eV, relatively akin to ZVD_Fe_Se@C_3_N_4_, indicating relatively weaker binding. This suggests that Se@C_3_N_4_ might not be the most suitable substrate for optimal drug delivery. Overall, the variations in adsorption energies across these systems highlight the importance of substrate selection in drug delivery applications. ZVD_Os_Se@C_3_N_4_ and ZVD_Ru_Se@C_3_N_4_ emerge as promising candidates, exhibiting stronger interactions with ZVD, while Fe_Se@C_3_N_4_ and Se@C_3_N_4_ display comparatively weaker binding, potentially impacting their suitability for efficient drug delivery. The pH-dependent drug release values further emphasize the need for a nuanced understanding of the environmental conditions in drug delivery systems.

**Table 7:** Adsorption energy and drug release analyses

Systems	*E*_complex_ (hartree)	*E*_adsorbate_ (hartree)	*E*_adsorbent_ (hartree)	Adsorption energy (eV)	BSSE (eV)	Drug release (a.u.)	Dipole moment (D)
ZVD_Fe_Se@C_3_N_4_	−6740.7	−5777.6	−963.1	−1.535	−1.561	−0.5	7.266
ZVD_Os_Se@C_3_N_4_	−5567.9	−4604.7	−963.1	−2.721	−2.679	−0.5	9.080
ZVD_Ru_Se@C_3_N_4_	−5572.1	−4608.9	−963.1	−2.721	−2.701	−0.5	10.047
ZVD_Se@C_3_N_4_	−5477.1	−4514	−963.1	−1.927	−1.945	−0.6	11.993

### 3.7 Drug release and pH

The investigation into the drug release mechanism from the adsorbents involved a comprehensive examination of the dipole moment and the influence of pH,^89^ aiming to shed light on the controlled release of ZVD. By analyzing the dipole moment and considering the impact of pH on the ZVD release from metal-doped graphitic carbon nitride nanocages, the study delved into the theoretical aspects of drug delivery in living systems. Firstly, the dipole moment was scrutinized to gain insights into the drug release process, as presented in Table 7. The dipole moment values for each system (ZVD_Fe_Se@C_3_N_4_, ZVD_Os_Se@C_3_N_4_, ZVD_Ru_Se@C_3_N_4_, and ZVD_Se@C_3_N_4_) were determined, providing a measure of the systems' polarity. These values, including 7.266 D for ZVD_Fe_Se@C_3_N_4_, 9.080 D for ZVD_Os_Se@C_3_N_4_, 10.047 D for ZVD_Ru_Se@C_3_N_4_, and 11.993 D for ZVD_Se@C_3_N_4_, indicate the distribution of charge within the systems, which is essential in understanding how drug molecules interact within them. Furthermore, the influence of pH on drug release was a critical aspect of the study, simulating the conditions encountered in the human body, particularly within the HIV cells with acidic pH environments.^90,91^ To account for this, the systems were protonated at the O atoms of ZVD with hydrogen, simulating an acidic environment, and re-optimized to understand the effects of increased acidity on drug release. The results indicated a pH-dependent drug release mechanism, crucial for controlled drug delivery. Analyzing the data, negative values in the drug release column (−0.5 and −0.6) suggest that drug release from these systems is favored under acidic conditions, such as those found in HIV cells. This implies that in acidic environments with lower pH, the drug remains slightly bound to the systems, increasing the likelihood of release. However, under more neutral or basic conditions, the drug release is favored, allowing for controlled and tailored drug delivery. Overall, the study's findings suggest that Os_Se@C_3_N_4_ and Ru_Se@C_3_N_4_ exhibit stronger interactions with the drug, potentially making them superior candidates for efficient drug delivery. The pH-dependent drug release mechanism highlights the potential for controlled drug release based on the environmental pH, providing opportunities for tailored drug delivery strategies, especially in contexts where pH variations play a crucial role in drug release kinetics.

### 3.8 Energy decomposition analysis (EDA)

Energy decomposition is a meticulous process that involves dissecting the overall energy of a system into its constituent components or contributing factors.^92^ This analytical approach provides a deeper understanding of how energy is distributed within the system, illuminating the specific elements that collectively constitute the total energy. By examining these individual parts, valuable insights into the underlying dynamics of the system can be uncovered, identifying the predominant energy sources, and fine-tune various aspects of the system to enhance its efficiency and overall performance.^93^ The system can be further divided into two fragments: ZVD and M_Se@C_3_N_4_, each with energy contributions acquired through the DFT B3LYP method. The total energy represents the comprehensive energy of the molecular system, which is the summation of all contributions within the system and mathematically expressed in eqn (3):

3 Δ*E*_tot_ = Δ*E*_int_ = Δ*E*_final_ − Δ*E*_A_ − Δ*E*_B_

A positive total energy signifies an unstable system characterized by low binding affinity and repulsive interactions, while a negative total energy signals a more stable system with a high binding affinity and strong attractive forces.^94^ In this analysis, all of the total energies are negative, indicating the stability of all interactions, as shown in Table S3 of the ESI† and Fig. 8. Notably, ZVD_Os_Se@C_3_N_4_ emerges as the most stable interaction, boasting the lowest total energy at −1837.9 kJ mol^−1^ compared to other compounds. This suggests that it exists in a more energetically favorable state than the rest. Osmium, a transition metal known for its resistance to corrosion and oxidation under most conditions, further supports the stability of this interaction. Interestingly, ZVD_Ru_Se@C_3_N_4_ and ZVD_Fe_Se@C_3_N_4_ exhibit the same total energy of −787.7 kJ mol^−1^, even though iron is typically more reactive than ruthenium under various conditions. This intriguing similarity in their total energy levels suggests that their stability is governed by factors beyond reactivity, possibly due to intricate orbital interactions. In contrast, ZVD_Se@C_3_N_4_ possesses a total energy of −262.6 kJ mol^−1^, making it the least stable among the complexes in terms of total energy. However, it is crucial to note that even with this lower stability, it is still considered a stable complex. The stability of a chemical complex depends not only on its total energy, but also on its specific interactions and electronic properties.^95^ The orbital energy of a complex reflects the cumulative impact of interactions between different molecular fragments within the system.^96^ Understanding the orbital energy is vital for deciphering the electronic transitions and orbital interactions responsible for the various components of the interaction energy.^97^ Notably, the orbital energy is directly proportional to the ionization potential, which plays a pivotal role in explaining how a drug delivery system can release drugs at specific sites. It is mathematically expressed in eqn (4):

4 Δ*E*_orb_ = final SCF Δ*E*_last_ − first SCF Δ*E*_first_

**Fig. 8:** Plots demonstrating the energy decomposition analysis (EDA) of the studied systems.

By examining the HOMO–LUMO table, it becomes evident that the complexes exhibit ionization potentials ranging from 5.812 to 6.502 eV. Specifically, ZVD_Fe_Se@C_3_N_4_ has an ionization potential of 6.104 eV, ZVD_Os_Se@C_3_N_4_ records 6.502 eV, ZVD_Ru_Se@C_3_N_4_ registers 6.109 eV, and ZVD_Se@C_3_N_4_ has the lowest ionization potential at 5.812 eV. To compare the ionization potentials with the orbital energies, we can assess the stability of various complexes. Notably, ZVD_Fe_Se@C_3_N_4_ stands out as the most stable complex in terms of its orbitals, boasting an impressively low orbital energy of −19691.3 kJ mol^−1^. This exceptional stability indicates that this complex holds a strong grip on its electrons, and is less likely to readily release them to a specific site. Conversely, ZVD_Se@C_3_N_4_ exhibits the least stability in terms of orbital interaction, with an orbital energy of −3150.6 kJ mol^−1^. While this energy level still reflects a stable state, it represents a significant contrast to the robust stability of ZVD_Fe_Se@C_3_N_4_. However, this contrast can be seen as an advantage because it implies that ZVD_Se@C_3_N_4_ is more predisposed to releasing electrons to a specific site. This characteristic is of paramount importance when considering drug delivery systems. The steric energy is the energy of the highest magnitude on our table, and is the difference of the orbital energy from the total energy as mathematically represented in eqn (5):

5 Δ*E*_steric_ = Δ*E*_tot_ − Δ*E*_orb_

In light of these observations, ZVD_Se@C_3_N_4_ once again emerges as the most promising candidate for the drug delivery of zidovudine. Its relatively moderate ionization potential, coupled with its willingness to release electrons, positions it as a prime candidate for targeted drug delivery applications, where controlled release of the drug payload is critical. This unique combination of stability and reactivity makes ZVD_Se@C_3_N_4_ an attractive option in the realm of pharmaceutical research and drug delivery technology.

### 3.9 Bond dissociation energies

Bond dissociation energies are a fundamental concept that plays a pivotal role in the understanding of chemical systems.^97^ This concept pertains to the amount of energy required to break the chemical bonds within a molecule, resulting in the conversion of those bonds into single atoms, smaller molecules, or even radicals. Such knowledge is essential for comprehending the stability and reactivity of compounds, which is especially valuable in the realm of chemistry and material science.^98^ In the analysis of these systems, various thermodynamic parameters are considered both before and after interaction with zidovudine, as presented in Table S4 of the ESI.† Among these parameters, enthalpy, which describes and characterizes the heat content or heat exchange involved in chemical and physical processes, stands out. Enthalpy is a critical factor as it helps us determine whether a given process is exothermic or endothermic. An exothermic process releases heat to the surrounding environment, resulting in a negative enthalpy value, while an endothermic process absorbs heat, yielding a positive enthalpy value.^98^ In this case, all of the systems exhibit negative enthalpy values, indicating that these systems are exothermic at both the surface and interaction levels. This means that these processes emit heat, contributing to the surroundings' thermal energy. Among the systems, ZVD_Fe_Se@C_3_N_4_ boasts the highest enthalpy values, both before and after interaction, with values of −5777.2 and −6740.0 hartrees, respectively. Following closely is ZVD_Ru_Se@C_3_N_4_, with an enthalpy of −4608.3 hartrees before interaction and −5571.1 hartrees after interaction. ZVD_Os_Se@C_3_N_4_ occupies the third position with an enthalpy of −4604.3 hartrees before interaction and −5567.1 hartrees after interaction, while ZVD_Se@C_3_N_4_ exhibits an enthalpy of −4513.6 hartrees before interaction and −5476.4 hartrees after interaction with the drug. Interestingly, the surface, represented by Fe_Se@C_3_N_4_, possesses a lower enthalpy of −5777.2 hartrees compared to the enthalpy of the interaction, which is −6740.1 hartrees. As known from thermodynamics, a lower enthalpy signifies a more stable state due to a lower internal energy. Therefore, the interaction of ZVD_Fe_Se@C_3_N_4_ is not energetically favorable compared to its surface counterpart. This trend continues with the rest of the complexes, such as ZVD_Ru_Se@C_3_N_4_, ZVD_Os_Se@C_3_N_4_, and ZVD_Se@C_3_N_4_, all displaying lower stability than their respective surface states. Hence, the order of enthalpy for the interaction is as follows: ZVD_Se@C_3_N_4_ < ZVD_Os_Se@C_3_N_4_ < ZVD_Ru_Se@C_3_N_4_ < ZVD_Fe_Se@C_3_N_4_. Moreover, the negative enthalpy values of these systems reveal that the reactants within each system possess higher internal energy compared to the products, reinforcing the exothermic nature of the interactions. In addition to enthalpy, another critical thermodynamic parameter to consider is entropy. Entropy measures the degree of disorder or randomness within a system.^99^ In this case, the entropy values increase from the surface to the interaction in the order of ZVD_Os_Se@C_3_N_4_ < ZVD_Se@C_3_N_4_ < ZVD_Ru_Se@C_3_N_4_ < ZVD_Se@C_3_N_4_. For the surfaces, entropy values typically range from approximately 200–215 cal mol^−1^-kelvin, whereas for the interactions, they increase to a range of 276–282 cal mol^−1^-kelvin. This escalation in entropy values underscores the increasing disorderliness or randomness within the systems as they transition from their surface states to the interaction with the zidovudine.

## 4 Conclusions

The electronic structure and energy distribution of materials used in sensing devices can be comprehensively understood through Density of States (DOS), which provides a detailed mapping of the energy levels accessible to electrons. This understanding is crucial in drug-delivery systems, such as the antiretroviral drug zidovudine (ZVD) used in HIV treatment. Specific drug molecules can alter DOS, leading to changes in the electronic properties of the material and affecting its conductivity. DOS is therefore an essential tool for understanding drug-delivery phenomena and optimizing delivery materials for enhanced sensitivity and selectivity. In this study, four systems incorporating ZVD_Fe_Se@C_3_N_4_, ZVD_Os_Se@C_3_N_4_, ZVD_Ru_Se@C_3_N_4_, and ZVD_Se@C_3_N_4_ were examined, and DOS helped elucidate the electronic structures and energy distribution profiles of the incorporated dopants. Fe emerged as a key element, shown in Fig. 4, with the ZVD_Fe_Se@C_3_N_4_ system having a relatively narrower energy gap of −0.4 to −0.6 eV, implying heightened reactivity, elevated conductivity, and amplified selectivity in delivering ZVD within the human body. Os introduced additional orbitals during the decoration process, which can facilitate mediating interactions with drug molecules and enhance the material's delivery capabilities. The study demonstrates the potential of the four systems, stimulated with Fe, Os, and Ru dopants, to advance drug delivery through tailored reactivity and conductivity. Visual studies, specifically the quantum theory of atoms-in-molecules (QTAIM), were also employed to study intramolecular and intermolecular interactions. QTAIM helps us understand interactions between molecules by analyzing bond critical points (BCPs) associated with quantum topological functions. Higher values of electron density (*ρ*(*r*)) indicate stronger chemical bonds, while lower values depict weaker chemical bonds. Negative values of Laplacian of electron density (∇^2^(*r*)) and potential energy density (*H*(*r*)) signify strong covalent interactions, positive ∇^2^(*r*) values and negative *H*(*r*) values indicate medium interactions, while both positive values (∇^2^(*r*) > 0, *H*(*r*) > 0) denote weak (non-covalent) interactions. Bonds attached to the drug carrier generally show medium interactions, except for specific bonds that indicate strong covalent interactions when interacting with the drug molecule. For example, bonds Se_54_–C_14_, Se_54_–C_6_, and Se_54_–O_5_ exhibit strong covalent interactions in the ZVD_Se@C_3_N_4_ complex. The study demonstrates that QTAIM is a valuable tool for understanding drug-delivery phenomena and optimizing delivery materials for enhanced sensitivity and selectivity. The electronic structure and energy distribution of materials used in sensing devices can be comprehensively understood through density of states (DOS), which provides a detailed mapping of the energy levels accessible to electrons. This understanding is crucial in drug-delivery systems, such as the antiretroviral drug zidovudine (ZVD) used in HIV treatment. Specific drug molecules can alter DOS, leading to changes in the electronic properties of the material and affecting its conductivity. DOS is therefore an essential tool for understanding drug-delivery phenomena and optimizing delivery materials for enhanced sensitivity and selectivity.

## Data availability

All other information regards to this study are presented in the ESI.†

## Author contributions

Hitler Louis: project conceptualization, design, resources and supervision. Favour A. Nelson: investigation, supervision, writing, analysis and manuscript first draft: Innocent Benjamin: visualization, analysis and writing. Rawlings A. Timothy: analysis, reviewing, writing, and editing.

## Conflicts of interest

All authors declare zero financial or inter-personal conflict of interest that could have influenced the research work or results reported in this research paper.

## Supplementary Material

RA-013-D3RA06885D-s001
